The article "The Theory of Planned Behavior for the Improvement of the Delayed Blood Donation Cycle, Optimization of the Planning Behavior, and Donor Intention" was retracted in 2023. Reasons: signs of a paper mill; compromised peer review; unreliable results or conclusions.

# The Theory of Planned Behavior for the Improvement of the Delayed Blood Donation Cycle, Optimization of the Planning Behavior, and Donor Intention

**DOI:** 10.1155/2022/3806431

**Published:** 2022-09-10

**Authors:** MinChuan Huang, IPing Chen, ShuYing Chung

**Affiliations:** ^1^School of Computer Science, Guangdong University of Petrochemical Technology, China; ^2^Institute of Nursing College, Central Taiwan University of Science and Technology, Taiwan

## Abstract

The advances in the technology applied to the health field lead the medical system to be optimized and the medical equipment and drugs to be improved, and the benefits can be seen in the prolonged human lifetime. The increased age and the lifestyle, however, increase the demand of blood for medical procedures and to save lives. The average age of blood donors has gradually increased, the number of new blood donors has grown slowly, and the allocation of blood supply and inventory is complex and many times cannot be improved. The low increase in blood donor number is a concern that needs to be overcome. Here, the theory of planned behavior was used as a tool to analyze the motivation, intention, and behavior of blood donors. The theory of planned behavior was applied in the form of questionnaires to college students. The results indicated that participation on the research motivates and educates the participants to donate blood, encourages the behavior of relatives, and leads the participants to realize the altruistic and mutually beneficial outlook on blood donation. The results also indicated the awareness of the students with respect to the importance of blood donation and that it can be an important tool in order to educate and increase the young blood donor number.

## 1. Introduction

COVID-19 has swept the world, with more than 168 million confirmed cases and more than 3.5 million deaths. Major disasters include the world's top ten military wars and terrorist attacks in 2020 [1, 2]. The development of artificial intelligence medical simulation teaching, new drug development, big data database, medical management information and communication technology, artificial blood research and development, and remote video medical system are urgent demands that need to follow the growth of the world population [3, 4].

In order to save lives and heal the wounded, the demand for blood is increasing day by day. So far, the research and development of artificial blood technology is difficult and the progress is slow [5–8]. The blood supply is insufficient and it is difficult to maintain its stability. According to the World Health Organization statistics in 2012, the median blood donation rate of high-income countries is 3.68%. If it reaches more than 5%, the blood can be completely self-sufficient. In 2015, the blood donation rate in Taiwan was 7.54%. The development of new strategies to improve the sources of blood for medical use represents a crucial demand, which would be desirable to be stable and uninterrupted. Strategic practices to develop and stabilize new blood sources and to encourage blood donation [9–11] include promoting the correct blood donation education, conveying the benefits of individual blood donation, promoting the concepts of friendship and mutual assistance and social responsibility, expanding fixed blood donation stations and itinerant blood donation vehicles, and conducting education lecture about blood donation at all communities and campus levels.

Among blood sources, human blood donation is the most consolidated practice to meet the clinical demand. In addition, the population of most countries is gradually aging, and the number of blood donors is decreasing, which is an irreversible and obvious problem. In an attempt to revert or at least to control this scenario, encouraging young people to donate blood can be seen as a promising alternative to overcome these concerns [12–14].

An important tool that can help to motivate young people to become new blood donors is the “theory of planned behavior” (TPB). Proposed by Icek Ajzen [15] and schematized in Figure 1, the theory preconizes that human behavior is the result of deliberate planning and is based on normative beliefs (beliefs influenced by the social pressures and perceived by the individual) and on control beliefs (beliefs that enable a behavior, under the control of the individual), which can understand the attitude and intention of behavior and can lead the behavior pattern to change, according to the perception of the behavior of the subject.

Attitude is the individual's positive or negative perception of behavior, evaluating a specific form of attitude after conceptualization. The composition of attitude is a function of an individual's significant belief in behavior outcome. Subjective norm is the social pressure that individuals feel when they take specific behaviors; the prediction of other people's behaviors has an influence on individual or group behavior decision-making and has an influence on individuals taking specific behaviors. Perceived behavioral control reflects the obstacles of personal past experience and expectation, and the more resources and opportunities available and the fewer obstacles expected, the stronger will be the perceptual behavior control. There are two ways of influence, which have motive meaning to behavior intention and can directly predict behavior. Attitude, the subjective norm and the perceived behavioral control, influences the behavior intention. It can be defined as the subjective probability of an individual taking a specific behavior that reflects the individual's willingness to take a specific behavior.

The behavior intention influences the behavior, which is defined as the act of an individual taking an action [15]. Considering the positive results of the application of the theory of planned behavior shown by many papers already reported in the literature, specifically on the attitude and behavior of college students' blood donation [16–21] (Table 1), this work aims to study the behavior patterns of this sample of students in an attempt to provide reference for blood donation planning units as a strategy to increase the number of young blood donors.

The application of the theory of planned behavior pattern aims to educate the students and can be considered to be socially relevant because it aims to widen the opportunity of saving lives and heal the wounded people who demand blood. The novelty of the study is the application of the theory in a limited young population composed of college students, a strategic age, and to educate them with the hope of increasing the number of blood donors in the future. The study is experimented by collecting questionnaires from college students followed by the evaluation of the responses. The questionnaires were prepared based on the principles of the theory of planed behavior, including the study of attitude, subjective norm, and perceived behavioral control and their influence on the behavior intention, which can finally influence the behavior.

## 2. Methods

### 2.1. Sample (Participants) and Design

The research was carried out using questionnaires applied to the students. In order to maintain the privacy and improve the college student's willingness to fill in the questionnaire, we have used the web to log in. The questionnaire was filled out anonymously and voluntarily. The web is called Wenjuanxing (http://www.wjx.cn). The information is filled in anonymously in order to protect the privacy of responders. SPSS statistical software was used for analysis. The participants were 113 students from the Department of Network Engineering, grade 2019, 89 boys and 24 girls.

### 2.2. The Questionnaires

The data collection was carried out by questionnaires designed by the authors. The questionnaires were prepared aiming to measure the motivation of the college students to donate blood, their blood donation experience, and behavior intention. A point scale was used in each case to analyze the responses.

The questionnaire analysis and achievement were based on the theoretical framework of planned behavior. We set up 12 unit items, including 6 questions of personal basic data, 9 questions of actual blood donation behavior, 4 questions of attitude, 4 questions of subjective norm, 3 questions of perceived behavior control, and 6 questions of behavior belief. The questionnaires were organized following the theory of planned behavior, as shown in Figure 2.

The questionnaires are presented in Section 3, with the respective responses and discussion. In short, 4 questionnaires were applied in order to understand the behavior of the students.

Questionnaire 1 collected personal data of the “Individuals” and “Analysis of social and economic background.” Questionnaire 2 was about blood donation experience and behavior intention. Questionnaire 3 was about the main variables of behavioral intention. Questionnaire 4 was about specificities of the variables of behavior intention. Questionnaires 1, 2, 3, and 4 and their respective responses are presented in Section 3.

### 2.3. Statistical Analysis

The data were used to determine the descriptive statistics such as percentages for gender, religion, ethnicity, and blood donation request and Shapiro-Wilk normality.

## 3. Results and Discussion

### 3.1. Individuals and Analysis of Social and Economic Background

The studied items were namely the class, gender, age, parents' education level, average monthly family income, parents' occupation, and the main sources of blood donation–related knowledge. The data are shown in Table 2. Age was an important data since young people are the main aim of this research. The age varied from 18 to 24 years, thus contributing to the reliability of the results that forward our objectives. The other social and economic aspects were variable, as can be seen in Table 2, contributing to the data variability.

### 3.2. Blood Donation Experience and Behavior Intention

The actual blood donation experience of the students was analyzed to highlight their beliefs and behavioral intentions.  Table 3 and Figure 3 show the results of the analysis of blood donation experience and behavior intention. The analyses showed that most of the participants (83%) have never donated blood, but if they have time, they were willing to be blood volunteers (80.5%). In addition, most of their relatives and friends (67.3%) have blood donation experience. These results reflected the personal experience and positive reinforcement of objects or behaviors—the greater the good impression, the stronger the perceptual behavior control of behaviors. The inner trust tends to the opinions and behaviors of family members, relatives, friends, and classmates around them, forming a bandwagon effect, which changes in the direction consistent with the majority of the group. The Shapiro-Wilk test showed a *p* value of 0.79, indicating that at the 0.05 level, the data was significantly drawn from a normally distributed population.

### 3.3. Analysis of the Main Variables of Behavioral Intention

Behavioral intention is determined by three main variables: behavioral attitude, subjective norm, and perceived behavioral control. The results shown in Table 4 and Figure 4 indicated that among the four types of attitude items, most of the students thought that blood donation was a good thing, and their attitude was in high agreement. Moreover, 96.5% and 91.2% of them thought that blood donation was worth doing, 87.6% of them thought that it is healthy, and 85% of them thought that it is safe. “In daily life, most of the people who are important to me think that I should donate blood, and they agree with me very much” reached up to 61.1%. Also, 64.6% of the patients supported blood donation. “For me, it was easy to donate blood” was 71.7%. “Whether I am willing to donate blood is up to me” is 95.6%. “As long as the blood bank needs me to donate blood, I can do it” reached 85%. The Shapiro-Wilk tests indicated that at the 0.05 level, most of the data was significantly drawn from a normally distributed population, as shown in Table 5. The one-sample *t*-test showed results for the parameters “very much agree, agree ordinary, disagree and very disagreeable,” with mean values 47.87 (±12.37), 31.70 (±3.33), 14.40 (±8.00), 4.66 (±4.55), and 1.37 (±1.65), respectively, showing that the population mean is significantly different, at the 0.05 level. The high percentage of “very much agree” and “agree” for attitude responses clearly suggests the behavior intention for blood donation, as evidenced in Figure 4. The objective norm and perceived behavioral intention also indicated that the participants can donate blood. In addition, it is possible to detect the valorization of the social behavior, which could be influenced by the theory of planned behavior learning, showing the efficiency of the strategy of its application in the education of the participants.

### 3.4. Analysis of Subdivided Variables of Behavior Intention

The three main variables that determine behavioral intention were subdivided into 7 more specific variables in order to deeply understand the student's behavior intention.  Table 6 and Figure 5 show the results of the analysis of the subdivided variables of behavior intention. Attitude included 6 questions of behavioral belief and 6 questions of outcome evaluation. Subjective norms included 5 questions of normative belief and 5 questions of conformity motivation. Perceptual behavior control included 7 items of control belief, 7 items of perceptual power, and 2 items of intention.

The results showed that most of the students think that blood donation can help people in need, and 100% of them agree with each other. Also, 98.2% of them believed that blood donation was a kind of mutually beneficial behavior. In addition, 85.8% of them were more confident of their own existence value, 21.2% of them lack a good feeling for blood donation pain, and 13.3% of them were worried that blood donation would expose their blood test report value. One-sample *t*-test showed that for the studied parameters “very much agree, agree ordinary, disagree and very disagreeable,” with mean values 29.93 (±16.79), 29.27 (±8.14), 27.64 (±12.34), 9.66 (±9.89), and 3.49 (±3.42), respectively, the population mean is significantly different at the 0.05 level.

The most common variables assigned as “very much agree” were “Blood donation can help people in need” followed by “Blood donation can extend the life of others” for 69.91 and 65.49% of the participants, respectively.

This study used the theory of planned behavior to educate college students and to explore the blood donation intention. The applied model studied the direct effects of attitude, objective norm, and perceived behavioral control on the intention to donate and the indirect influence of behavior belief, normative belief, perception, and others on blood donation intention. These results represent an important parameter to predict and encourage the social actions related to blood donation and can be used for the construction of plans for this specific field of public health. The data resulting from the analysis of the responses provide support for understanding the variables that are relevant to blood donation within this specific young studied population.

In general, the results showed that most scholars believe that personal social, economic, and cultural backgrounds, such as personality, intelligence, experience, age, gender, and cultural background, affect behavioral beliefs and attitudes, subjective norms, and perceived behavioral control, and ultimately affect behavioral intention and behavior. Behavioral attitude, subjective norm, and perceived behavioral control are the three main variables that determine behavioral intention. The more positive the attitude is, the stronger the perceived behavioral control is and the greater the behavioral intention of the individual, and sociocultural factors (personality, intelligence, experience, age, gender, and cultural background) indirectly affect behavior attitude, subjective norms, and perceived behavior control, and ultimately affect behavior intention and behavior.

In some European countries, the national blood donation rate is more than 5%, and the blood can be self-sufficient. The slogan of the World Blood Donor Day in 2019 is “safe blood for all.” According to the report on global blood safety and supply issued by the World Health Organization, the number of unpaid blood donors and the amount of blood collected in China rank the first in the world. There are 32 blood centers, 321 central blood stations, 99 central blood banks, and 1390 fixed blood collection points in China. The blood donation rate was increased from 4.8‰ in 1998 to 11‰ in 2017. The number of unpaid blood donors was 14.59 million in 2017, and the total amount of blood donation reached 4956 tons [14, 22, 23].

These data indicate that it is necessary to increase the number of young first-time blood donors in order to supply the future demand for the clinical use of blood. In this vein, the research performed by the scholars all over the world can be a potential tool to increase blood donation once it can encourage these scholars. The research evidenced the implicit knowledge of college students about blood donation, evaluation of their blood donation knowledge, understanding of their blood donation attitude, and practicing of blood donation behavior [9, 12, 24, 25] and also can educate, encourage, and motivate them for blood donation. The most important result found here was that shown in Table 4 and Figure 4, with respect to the main variables of behavioral intention, in which most of the responses were “very agree” and “agree” for the intention of blood donation, reaching percentages around 67 and 30% for “very much agree” and “agree,” respectively, for the question “I think blood donation is a good thing.” The mean values for “very much agree” and “agree” were about 47.87 and 31% considering all the studied parameters of attitude, objective norm, and perceived behavior control, indicating that the intention to donate blood is high in this specific population.

With respect to the responses to the subdivided variables of behavior intention, parameters were more dispersed, as expected, because of the very specific questions, including the question about normative beliefs and control beliefs, among others, which can trigger the worry about the priorities. Nonetheless, the responses for “very much agree” and “agree” were 30 and 29%, almost 60% in total, indicating the positive tendency to donate blood.

The credit system of quality education in colleges and universities is one of the requirements for graduates. They must accumulate 4 credits. Quality development is the concrete expression of thought and behavior in school life. It includes academic technology and professional skills, cultural arts and sports competitions, social practice, and voluntary service. We should improve the cultural taste of college students, strengthen social responsibility and vocational education, and improve their aesthetic taste and humanistic quality. Voluntary blood donation is also included in this project, which can get 0.2 points, which is helpful for college students' willingness to donate blood [26, 27].

In addition, qualitative interviews with senior nurses in blood donation units for more than 10 years showed that all nurses had professional qualification certificates and rich experience in blood collection. Regular blood donation between schools and public service units is the most cooperative. Combined with the auspicious celebration activities close to the society, the incentive effect of civil society organizations using daily necessities and livelihood materials is the biggest. The mobile app clustering software is used to make blood donation appointments, provide feedback on personal blood test data, remind the time and place of the activity, timely display blood donation photos and videos, and achieve the best adhesion and reaction with blood donors, forming the flying-geese model and conformity psychology.

The popularization of the Internet and the sharing of mobile applications improved the research quality once the application of questionnaires can be used for large groups. The use of the theory of planned behavior can be useful to educate and expand the young blood donation groups; encourage students to participate in the blood donation knowledge competition; learn the correct blood donation knowledge; understand students' blood donation intention and planned behavior; maintain self-qualified blood donation conditions; expand young people's willingness to donate blood; encourage the behavior of relatives, friends, and classmates; and join the blood donor group and also realize the altruistic and mutually beneficial outlook on blood donation.

## 4. Conclusions

Every college student has a large number of different types of behavioral beliefs during their study. Only a small number of behavioral beliefs are prominent beliefs, which are touched in a specific time and environment. These prominent beliefs are related to behavioral attitude, subjective norms, and perceived behavioral control. Blood donation has independent cognition, common belief, and social emotional foundation. Individuals' original family and social culture affect the behavior belief and also indirectly affect the behavior attitude, subjective norms, and perceived behavior control, ultimately affecting the blood donation behavior intention and actual behavior. The results of the main variables of behavioral intention, in which most of the responses were “very agree” and “agree” for the intention of blood donation, reached percentages of about 67 and 30% for “very much agree” and “agree,” respectively, for the question “I think blood donation is a good thing.” The mean values for “very much agree” and “agree” were about 47.87 and 31%, considering all the studied parameters of attitude, objective norm, and perceived behavior control, indicating that the intention to donate blood is high in this specific population. The results of the subdivided variables of behavior intention parameters were more dispersed, as expected, because of the very specific questions, including the question about normative beliefs and control beliefs, among others, which can trigger the worry about the priorities; however, they also indicated high tendency to donate blood.

## Figures and Tables

**Figure 1:** Theory of planned behavior.

**Figure 2:** The questionnaire project diagram of the theory of planned behavior.

**Figure 3:** The results of blood donation experience and behavior intention.

**Figure 4:** The results of the analysis of the main variables of behavioral intention: (a) attitude, (b) objective norm, and (c) perceived behavioral control.

**Figure 5:** Results of the subdivided variables of behavior intention.

**Table 1:** Samples of the use of theory of planned behavior to study the intention of the students to perform blood donation, showing the sample and the main results.

Sample	Results	Reference
Students at a public higher learning institution in Malaysia	The results showed that knowledge that the more blood they donate, the more lives will be saved influences the students' intention to blood donation	[18]
Private higher education students, Jimma town, Oromia, Ethiopia	Blood donation intentions are mainly determined by perceived barriers, subjective norms, and the attitude of respondents toward voluntary blood donation	[19]
Undergraduate students at the University of Ulster, Coleraine	The results provided strong support for the role of self-efficacy as a major determinant of blood donation intention	[20]
Medical students in Pakistan	The results indicated that perceived behavioral control, anticipated regret, and attitude were the most influential factors in determining intention of blood donation	[16]
University students, 18 years or older, since this is the minimum age necessary to give blood	The results indicate that self-efficacy is the construct with the greatest influence on the intention to donate blood, followed by attitude, with moral norm also having a high indirect influence through attitude	[21]
Undergraduate students at College of Health Sciences in Northeast Portugal	The results showed that the motivations of “be a civic duty” had a significant impact on donor status	[17]

**Table 2:** Analysis of social and economic background.

Distinguish	Content description
Class	There are 113 students in the department of network engineering, grade 2019
Gender	78.8% boys and 21.2% girls
Age	There were 0.9% person aged 18, 10.6% persons aged 19, 38.9% persons aged 20, 37.2% persons aged 21, 11.5% persons aged 22, and 0.9% person aged 24
Parents' education level	There were 54.9% below junior middle school, 30.1% at senior middle school, 15% at junior college and university, and 0 person above master's degree
Average monthly household income	69% have an average monthly income of less than 10000 yuan (including), 19.5% have an average monthly income of 10001–15000 yuan, 7.1% have an average monthly income of 15001–20000 yuan, and 4.4% have an average monthly income of 20001–30000 yuan
Parent occupation	7.1% were government officials, 3.5% were businessmen, 29.2% were workers, 21.2% were farmers, 5.3% were doctors, 5.3% were service workers, 20.4% were self-employed, 0.9% were family managers, 2.7% were unemployed, and 9.7% were others
The main sources of blood donation–related knowledge	83.2% were mobile phone and internet users, 9.7% were roommates, 5.3% were relatives, and 1.8% were others

**Table 3:** Analysis of blood donation experience and behavior intention.

	Content description	
Distinguish	Yes	No
Have you ever offered blood?	55 (48.7%)	58 (51.3%)
Are you willing to donate blood regularly (every 2–3 months when you can do so)?	31 (27.4%)	82 (72.6%)
Have you ever offered platelets?	9 (8%)	104 (92.0%)
Are you willing to donate platelets regularly (every 2–3 weeks when platelets are available)?	62 (54.9%)	51 (45.1%)
Have you ever been a blood donor?	19 (16.8%)	94 (83.2%)
If you have time, are you willing to be a blood volunteer?	91 (80.5%)	22 (19.5%)
Have you ever received the certificate of honor related to blood donation?	27 (23.9%)	86 (76.1%)
Have you ever received any souvenirs or gifts related to blood donation?	55 (48.7%)	58 (51.3%)
Do your relatives and friends have blood donation experience?	76 (67.3%)	37 (32.7%)

**Table 4:** Analysis of the main variables of behavioral intention.

		Response (%)				
Distinguish	Content description	Very much agree	Agree	Ordinary	Disagree	Very disagreeable
Attitude	I think blood donation is a good thing	67.26	29.20	3.54	0.00	0.00
	I think it's worthwhile for me to donate blood	61.95	29.20	7.96	0.88	0.00
	I think it's healthy for me to donate blood	53.98	33.63	9.73	2.65	0.00
	I think it's safe to donate blood	52.21	32.74	14.16	0.88	0.00
Objective norm	In my daily life most people who are important to me think that I should donate blood	34.51	26.55	22.12	14.16	2.65
	In my daily life most of the people who are important to me support me to donate blood	37.17	27.43	23.89	8.85	2.65
	In my daily life most important groups think I should donate blood	34.51	30.09	24.78	6.19	4.42
	In my daily life most important groups support me to donate blood	37.17	35.40	22.12	4.42	0.88
Perceived behavioral control	It's easy for me to donate blood	37.17	34.51	15.04	9.73	3.54
	It's up to me whether I want to donate blood or not	61.95	33.63	2.65	1.77	0.00
	As long as the blood bank needs me to donate blood, I can do it	48.67	36.28	12.39	1.77	0.88

**Table 5:** Results of the normality test.

	Statistic	*p* value
Very much agree	0.8707	0.07915
Agree	0.93283	0.44015
Ordinary	0.92149	0.33127
Disagree	0.87848	0.09952
Very disagreeable	0.8097	0.01262

**Table 6:** Analysis of subdivided variables of behavior intention.

Distinguish	Content description	Very much agree	Agree	Ordinary	Disagree	Very disagreeable
Behavior belief	Blood donation can help people in need	69.91	30.09	0.00	0.00	0.00
	Blood donation can extend the life of others	65.49	32.74	0.88	0.88	0.00
	I think blood donation is a mutually beneficial act	57.52	26.55	9.73	5.31	0.88
	Blood donation makes me sure of my value	53.10	32.74	10.62	2.65	0.88
	The pain of blood donation is lack of favor	8.85	12.39	40.71	29.20	8.85
	I'm worried that blood donation will expose my blood test report value	7.96	5.31	37.17	35.40	14.16
Result evaluation	I can accept blood donation. Blood donation can help people in need	58.41	34.51	7.08	0.00	0.00
	I can accept blood donation. Blood donation can extend the life of others	60.18	33.63	5.31	0.88	0.00
	I can accept blood donation. I think it's a mutually beneficial act	56.64	30.09	9.73	2.65	0.88
	I can accept blood donation. Which makes me sure of my value	53.98	35.40	8.85	1.77	0.00
	Blood donation is painful. I do not like blood donation	14.16	6.19	31.86	37.17	10.62
	I accept blood donation even if it may expose my blood test report value	18.58	18.58	30.97	20.35	11.50
Normative belief	My “close male (female) friend” thinks I should donate blood	22.12	29.20	38.05	6.19	4.42
	My parents and family elders think I should donate blood	21.24	27.43	37.17	8.85	5.31
	My brothers and sisters think I should donate blood	23.01	29.20	38.05	6.19	3.54
	My classmates and friends think I should donate blood	26.55	30.97	36.28	4.42	1.77
	My “paramedics” think I should donate blood	30.97	29.20	31.86	5.31	2.65
Subordinate motive	I will be encouraged to donate blood because of my intimate male (female) friends	28.32	30.97	35.40	3.54	1.77
	I would donate blood on the advice of my parents and family elders	26.55	33.63	34.51	4.42	0.88
	I will donate blood because of my “brothers and sisters” suggestion	24.78	33.63	36.28	4.42	0.88
	I will donate blood because of “classmates, friends” suggestions	23.01	29.20	38.94	7.08	1.77
	I will give blood on the recommendation of “medical staff”	23.89	34.51	34.51	6.19	0.88
Control beliefs	“Too busy studying or working” will make me not want to donate blood	14.16	22.12	30.97	28.32	4.42
	“Inconvenient traffic” will make me not want to donate blood	13.27	25.66	27.43	27.43	6.19
	Because “do not understand the conditions of blood donation” will make me not want to donate blood	14.16	29.20	27.43	23.01	6.19
	My encouragement from friends and relatives will give me blood	23.01	33.63	31.86	9.73	1.77
	“Holidays, work holidays” will make me want to donate blood	15.93	35.40	38.05	7.96	2.65
	I think I have enough blood to donate	22.12	41.59	21.24	8.85	6.19
	I went to donate blood because “someone in the family needs blood transfusion”	32.74	37.17	24.78	4.42	0.88
Perception	“Too busy at school or work” I still want to donate blood	20.35	30.97	37.17	7.96	3.54
	“Blood donation location is not convenient” I still want to donate blood	21.24	26.55	39.82	8.85	3.54
	I still want to donate blood if I do not understand the conditions of blood donation	22.12	20.35	41.59	11.50	4.42
	“Friends and relatives” do not encourage me to donate blood	19.47	28.32	39.82	6.19	6.19
	I will arrange “holiday, work leave” to donate blood	21.24	39.82	30.09	5.31	3.54
	I believe that my physical condition is suitable for blood donation	29.20	41.59	19.47	5.31	4.42
	I think blood donation is a kind of mutually beneficial behavior and a concept of reserve	37.17	37.17	23.01	2.65	0.00
Intention	I will regularly donate blood in the next year	22.12	27.43	33.63	11.50	5.31
	I would like to participate in blood donation activities held by all organizing groups and units	33.63	29.20	30.09	5.31	1.77

## Data Availability

The data used to support the findings of this study are available from the corresponding author on request.
